RETRACTED

# The analysis of the influence of fractal structure of stimuli on fractal dynamics in fixational eye movements and EEG signal

**DOI:** 10.1038/srep26639

**Published:** 2016-05-24

**Authors:** Hamidreza Namazi, Vladimir V. Kulish, Amin Akrami

**Affiliations:** 1 School of Mechanical and Aerospace Engineering, Nanyang Technological University, Singapore; 2 School of Mechanical engineering, University of Tehran, Iran

## Abstract

One of the major challenges in vision research is to analyze the effect of visual stimuli on human vision. However, no relationship has been yet discovered between the structure of the visual stimulus, and the structure of fixational eye movements. This study reveals the plasticity of human fixational eye movements in relation to the ‘complex’ visual stimulus. We demonstrated that the fractal temporal structure of visual dynamics shifts towards the fractal dynamics of the visual stimulus (image). The results showed that images with higher complexity (higher fractality) cause fixational eye movements with lower fractality. Considering the brain, as the main part of nervous system that is engaged in eye movements, we analyzed the governed Electroencephalogram (EEG) signal during fixation. We have found out that there is a coupling between fractality of image, EEG and fixational eye movements. The capability observed in this research can be further investigated and applied for treatment of different vision disorders.

Eye-movement refers to the voluntary or involuntary movement of the eyes, helping in acquiring, fixating and tracking visual stimuli. While we fixate our gaze, the eye movements drive our visual experience. In fact, our visual system has a built-in contradiction: when we direct our gaze at an object of interest, our eyes are never still. Therefore the analysis of perception, physiology, and computational modelling of fixational eye movements is critical to our understanding of vision in general, and also to the understanding of the neural computations that work to overcome neural adaptation in normal subjects as well as in clinical patients.

For a long time, phenomena which do not have a regular or predictable pattern tended to be ignored and not worthy to study. But, it is now found that irregular patterns can provide adequate explanations for many natural phenomena. Fractal theory is proposed to study these irregular patterns. Nowadays, it is common knowledge that fractal phenomena are ubiquitous in nature. Since Mandelbrot^1^ showed self-similarity properties in geometry, scientists in different fields have tried to apply the fractal theory in order to explain irregular and apparently ambiguous patterns and many articles have been published indicating fractal properties. Fractal dimension is a measure used to quantify fractal patterns. In fact, fractal dimension can be viewed as an index of complexity, which shows how a detail in a pattern changes with the scale at which it is measured.

RETRACTED

Although, in medical science, fractal properties have been reported for various cases such as DNA^2^, Blood vessel and pulmonary vessels^3^, heart sound^4^, heart rate^5^, EEG signal^6^, bone structure^7^ and human stride time series^8^, there have been limited works which analyzed the fractal dynamics of eye movements as a random walk. Besides some works which found out the fractal nature of fixational eye movements^9^,^10^, some scientists have worked on analysis of eye movements in healthy or unhealthy subjects. Some of these works considered the fractal analysis of eye movements without considering the fractal structure of visual stimuli. For instance, Schmeisser *et al*.^11^ analyzed the eye movements of normal and abnormal readers for evidence of chaotic, nonlinear dynamical behaviour. Based on their results, the computed fractal dimension of the system’s presumed attractor directly related to qualitative assessment of reading ability. In another work, Belyaev *et al*.^12^ analyzed the fractal dimension of eye movements of subjects while they were looking at different images. The results of their study showed that the fractal dimension of trajectory of eyes movement in small degree depends on image type, and also on an f angle of its vision. Also, it was shown that the fractal dimension strongly changes depending on the specific observer, and also from a type of the eyes movements (fixings or saccades). Also look at^13^,^14^,^15^. Some studies analyzed the eye movements without considering its fractal dynamics, but focusing on fractal structure of visual stimulus. For instance, Nagai *et al*. investigated the relationship between the gaze location and fractal dimension of visual stimulus. Their analysis showed that fractal dimension was higher for those areas where gaze was concentrated than for other areas^16^. In a recent study Marlow *et al*. investigated the dynamic structure of human gaze over time during free viewing of computer-generated fractal images using the Hurst exponent. They found out that the Hurst exponent was invariant across all participants, including those with distinct changes to higher order visual processes due to neural degeneration^17^. Wu *et al*.^18^ analyzed the temporal dynamics of eye movements for subjects who were looking at scenes with different fractal dimensions. They found out that temporal dynamics of eye movements were related to differences in scene complexity and clutter. Also look at^19^. Based on all these studies, stimuli have a powerful draw on the allocation of subjects’ eyes attention.

RETRACTED

Beside all works on this area of research, the effect of fractal content of stimulus on fractal dynamics of eye movements and EEG signal has not been investigated yet. In this paper, we propose a novel analysis in order to reveal the effect of structural features of the visual stimuli on human vision. Particularly, we indicate that how fractal structure of a visual stimulus plays significant role on fractal dynamics of eye movements. First, we examine fractal dimensions of some pictures. Then, we record eye movements and EEG signals of subjects while looking at pictures, and analyze their fractal exponents. We analyze the coupling between the fractal structure of stimulus and eye movements by linking it to the nervous system. Finally, discussion and recommendation will be drawn.

## Method

Eye movements in looking at different patterns or reading can be idealized as an alternating sequence of fixations and saccades that move through visual stimuli in discrete steps. When we watch a scene, fixation duration and saccade length vary greatly. Considering that fixation duration and saccade length are random variables generated by an underlying stochastic process, the goal of this study was to analyze the effect of fractal structure of visual stimulus on fractal dynamics of human fixational eye movements. Based on Fig. 1, tremor, drift, and micro saccades are different components of fixational eye movements^20^,^21^,^22^. Physiological drift and micro saccades are the two most important components of fixational eye movements. Physiological drift is a slow random component that could be characterized as a diffusion process. Micro saccades are rapid small-amplitude movements. Tremor is a small-amplitude, oscillatory component superimposed to drift.

We have used three visual stimuli with different fractal exponents. These stimuli were Apollonian gasket, Sierpinski Hexagon and Penrose tiling. We computed the fractal dimension for each stimulus using a MATLAB based code that we have written. This code computes the fractal dimension based on box counting method^23^.

We asked the subjects to look at each stimulus, and analyzed the fractal structure of their resultant eye movement time series to determine its relation with the stimuli used. In order to explain the eye movements by linking it to the nervous system, we also collected the EEG signals of subjects in this experiment. This analysis was due to the fact that eye movements appear to be initiated by a small cortical region in the brain’s frontal lobe. Also, the brain is engaged in perception of stimuli. A schematic of the experimental design is presented in Fig. 2.

RETRACTED

Based on this methodology, we concurrently collected eye movements and EEG signal and then analyzed their fractal property by computing the fractal dimension.

### Data collection

In this research the experiments were carried out on 60 voluntary healthy students, 30 males and 30 females with the age of 22–24 years old, with normal vision (without any vision problem). The subjects never wore glasses. Prior to the experiment, each subject was examined and interviewed by a physician to ensure no vision problem, neurological deficit, pain condition, or medication affects the vision or EEG data collection. The nature of study was explained to participants before the experiments and then the written informed consent was obtained from them. All procedures were approved by the Internal Review Board of Nanyang Technological University and the approval for experimentation involving human subjects was issued by the university. The study was carried out in accordance with the approved guidelines. It is noteworthy that the identity of all subjects remains confidential.

In an electrically shielded, acoustically isolated and dimly illuminated room, three visual stimuli with different fractal dimension were applied on subjects and we asked them to view each photograph as they would normally look at scenes. The visual stimuli are shown in Fig. 3. In this figure, the third stimulus (Penrose tiling) has a bigger fractal dimension than the second stimulus (Sierpinski Hexagon), which itself has a bigger fractal dimension than first stimulus (Apollonian gasket). It should be mentioned that it was endeavoured to insulate the subjects from all other external stimuli. This ensures that the response measured in the eye movement and EEG signals is primarily due to the stimulus applied.

We used an Eyelink 1000 (SR Research, Ottawa, ON, Canada) eye-tracking system in order to record participants’ eye movements at 1000 Hz. The images, with the size of 768 × 768 pixels, were presented to participants on the monitor of a computer from 60 cm distance. The images were subtending the vertical and horizontal visual angles of 24°. The participants looked at the computer monitor while with their heads positioned in a chin rest.

The EEG data used in this research were collected using Mindset 24 device, a 24-channel topographic neuro-mapping instrument, which measures 24 channels of data. In this research, the electrode impedance was kept lower than 5 KΩ and the sampling frequency was 256 Hz. Mindmeld 24 software was used for the collection of data using Mindset 24 machine. The software gives data in the form of .bin files which can be processed to give text files (.txt) that are required for further processing.

RETRACTED

At first, eye movements and EEG signals were collected for 3 seconds in non-stimulus condition while the monitor showed the white screen. Then, the first stimulus appeared on the computer screen for 3 seconds and then it disappeared and the white screen appeared. This trend was continued for the second and third stimuli with inter-stimulus interval of 10 seconds. It should be mentioned that a bipolar electrooculogram (EOG, vertical and horizontal) was recorded for off-line artifacts rejection.

In the first day 5 trials were collected in case of each stimulus from each subject. The data collections were repeated in the second day for each subject in order to examine the reproducibility of the results from experiments. By repeating the experiments in the second day, a total of 10 trials were collected in case of each stimulus from each subject for further analysis. It is noteworthy that physician monitored the subjects during all experiments.

### Data analysis

Raw eye-movement data were pre-processed using a program written in MATLAB by removing fixations that occurred around eye blinks or outside the presentation screen. Only distracted fixations and the two adjacent non-distracted fixations (served as baseline) were processed further. This program then generated the filtered eye movements time series and computes its fractal dimension.

In case of analysis of EEG data, as the recorded data were noisy, at first the EEG signals were filtered using Wavelet toolbox in MATLAB and then were processed for computing of fractal dimension. It should be mentioned here that, although EEG data were recorded from 24 electrodes, the analysis was done on the data governed from the left occipital (O1) electrode (near to the location of the visual primary sensory area). This electrode was chosen based on the nearest place to the visual sensory area which shows the strongest response that can be seen in the signal recorded from this electrode compared to other electrodes.

It is noteworthy that computation of fractal dimension in case of eye movement time series and EEG signal was based on the box counting method^6^.

It should be mentioned that all subjects and all trials were included in the analysis. The data were inspected for differences between right and left eyes using statistical analysis.

### Statistical Analysis

Mean values for the dependent variables –fractal scaling exponent of fixational eye movements– were compared across visual stimulus and no stimulus conditions with a one-way repeated measures ANOVA. Mauchly’s test (*α* = 0.05) was implemented to test for sphericity. In fact, Mauchly’s sphericity test is a statistical test used to validate a repeated measures analysis of variance (ANOVA). As another statistical test, post-hoc test was run to confirm where the differences occurred between groups (multiple comparisons). Trend analysis was performed across conditions when ordered according to the fractal properties of the visual stimuli e.g. increasing the fractal exponent from the first to the third image. For a repeated measures design, we used Omega squared (*ω*^2^) as an unbiased measure of effect size suitable for small samples; In order to do pairwise comparisons effect size, *r*, was used. All statistical analyses were performed using SPSS software. It is noteworthy in order to have robust results, all assumptions in case of each statistical test were fulfilled.

RETRACTED

## Results

We conducted Two-sample Kolmogorov–Smirnov test with 95% confidence level in order to test the governed data from right and left eyes. As the result of the test indicated that the data for the right and left eyes are not different, here we report the results for the right eye.

Mauchly’s test indicated that the assumption of sphericity had not been violated. There was a significant effect of the visual stimulus on the fractal exponent of the fixational eye movements (*P* < 0.05), with an effect size *ω*^2^ = 0.86. In general, the application of the visual stimulus reduced the fractal dimension of fixational eye movements. A significant linear trend between visual stimulus conditions was observed (*P* < 0.05), indicating that the third stimulus (Penrose tiling) yielded a bigger change in the fractal dimension of fixational eye movements than the second stimulus (Sierpinski Hexagon), followed by the first stimulus (Apollonian gasket), mirroring the trend in fractal properties of the visual stimulus themselves i.e. the third stimulus bigger than the second stimulus, bigger than the first stimulus (Fig. 4). The effect size calculations between different conditions suggest that the third stimulus led to the greatest change in the fractal exponent of fixational eye movements with large effect sizes (r > 0.5) observed across all Penrose tiling comparisons (Table 1).

As mentioned before, eye movements are initiated by a small cortical region in the brain’s frontal lobe and then brain precepts the stimulus. Thus, the observed trend in fixational eye movements should be related to the EEG signal. In other words, there should be a coupling between fractal properties of visual stimulus, EEG signal and eye movements. In order to test this coupling and explain the behaviour seen in Fig. 4, we bring the results of analysis of EEG signals in Fig. 5.

RETRACTED

Based on Fig. 5, similarly there was a significant effect of visual stimulus on the fractal exponent of the EEG signal (*P* < 0.05), with an effect size *ω*^2^ = 0.76. A significant linear trend between visual stimulus conditions was observed (*P* < 0.05), indicating that the third stimulus yielded a bigger change in the fractal dimension of the EEG signal than the second stimulus, followed by the first stimulus, mirroring the trend in fractal properties of the visual stimulus themselves i.e. the third stimulus bigger than the second stimulus, bigger than the first stimulus. Effect size calculations between conditions suggest that the third stimulus led to the greatest change in the fractal exponent of the EEG signal with large effect sizes (r > 0.5) observed across all Penrose tiling comparisons (Table 1).

The behaviour seen in our analysis can be explained through information theory. The image with a higher fractal dimension contains more information which accordingly transferred to the brain due to stimulation. The Hurst exponent which is indicator of the memory of the system can be discussed here. The Hurst exponent (H) is a statistical measure used to classify time series. The Hurst exponent can have any value between 0 and 1. If the Hurst exponent has a value between 0 and 0.5, it means that the process is anti-persistent i.e. the trend of the value of the process at the next instant will be opposite to the trend in the previous instant. Secondly, a value of H between 0.5 and 1 means that the process is persistent i.e., the trend of the value of the process at the next instant will be the same as the trend in the previous instant. Finally, If H = 0.5, the process is considered to be truly random (e.g., Brownian motion). It means that there is absolutely no correlation between any values of the process. We have shown before that as information is transferred to the brain in any form of stimulation, the value of the Hurst exponent increases^24^. In other words, the brain memory increases due to stimulation. If more information is transferred to the brain, we will have a bigger increment in the value of the Hurst exponent. On the other hand, increasing the value of the Hurst exponent will cause decreasing of the complexity of the signal which is mapped on decrement of its fractal dimension^6^. So, it is clear that by choosing the stimulus that is more fractal and contains more information, we will see a bigger reduction in EEG signal fractal dimension.

It is noteworthy that, based on the effect size analysis, the visual stimulus had a bigger effect on the fractal dynamics of eye movements than the EEG signal. This is due to the fact that the stimulus has a bigger effect on eye movements and less effect on EEG signals. In other words, when we look at an image, our eyes process all parts of the image, but they will only send a message to the brain about those parts of the image that are more important to us (bigger than the threshold stimulus), and accordingly will cause perception. In summary, an adaptation occurred in the EEG signal and eye movements’ dynamics as a result of looking at visual stimuli.

RETRACTED

## Discussion

In this paper we analyzed the effect of fractal property of visual stimuli on fractal dynamics of human fixational eye movements. In order to explain the eye movements by linking it to the nervous system, we also analyzed the EEG signals of subjects. Our findings demonstrated plasticity of the visual-motor phenomenon during looking at visual stimuli, as the trend across the fractal structure of visual stimuli is mirrored in the trend across the reduction of fractal exponent of EEG signal and fixational eye movements. It was shown that the third stimulus with a higher value of fractal dimension caused a bigger change in the fractal exponent of the EEG signal and fixational eye movements, compared to the second and first stimuli. This behaviour was seen in comparison between the second and first stimuli as well. Based on the results the EEG signal was affected less than eye movements due to stimulation.

The method discussed in this research can be further applied in case of patients with some vision diseases that deteriorate their eye movements focus, in order to study the fractal behaviour of fixational eye movements in case of different fractal visual stimuli. Based on the result of analysis, scientists could be able to advise on proper visual stimuli in order to improve the patient’s vision. On the other hand, developing a mathematical model which makes a link between the fractal properties of visual stimulus and the fixational eye movements can be investigated. This model can be developed based on our recent fractional diffusion model of EEG signals which was developed in^24^. This model can be well employed for further investigations in vision science and engineering.

## Additional Information

**How to cite this article**: Namazi, H. *et al*. The analysis of the influence of fractal structure of stimuli on fractal dynamics in fixational eye movements and EEG signal. *Sci. Rep.* **6**, 26639; doi: 10.1038/srep26639 (2016).

## Figures and Tables

**Figure 1:** Example of fixational eye movements.

**Figure 2:** A schematic of the experiment.

**Figure 3:** Three visual stimuli (with their fractal dimension) applied on subjects.

RETRACTED

**Figure 4:** Fractal dimension of the visual stimuli is shown on the right for illustration purposes. Fractal analysis of the fixational eye movements across different stimuli, for all subjects, is shown on the left. Error bars are standard deviations.

**Figure 5:** Fractal analysis of the EEG signals across different stimuli, for all subjects. Error bars are standard deviations.

**Table 1:** Effect sizes for pairwise comparisons.

Condition	Eye movement’s fractal dimension	EEG signal’s fractal dimension
	Effect size (*r*)	Effect size (*r*)
No stimulus vs. Apollonian gasket	0.83	0.78
No stimulus vs. Sierpinski Hexagon	0.90	0.92
No stimulus vs. Penrose tiling	0.96	0.93
Apollonian gasket vs. Sierpinski Hexagon	0.58	0.49
Apollonian gasket vs. Penrose tiling	0.89	0.74
Sierpinski Hexagon vs. Penrose tiling	0.79	0.58
